# Score and Correlation Coefficient-Based Feature Selection for Predicting Heart Failure Diagnosis by Using Machine Learning Algorithms

**DOI:** 10.1155/2021/8500314

**Published:** 2021-12-20

**Authors:** Ebrahim Mohammed Senan, Ibrahim Abunadi, Mukti E. Jadhav, Suliman Mohamed Fati

**Affiliations:** ^1^Department of Computer Science & Information Technology, Dr. Babasaheb Ambedkar Marathwada University, Aurangabad, India; ^2^Information Systems Department, Prince Sultan University, Riyadh, Saudi Arabia; ^3^Shri Shivaji Science & Arts College, Chikhli Dist., Buldana, India

## Abstract

Cardiovascular disease (CVD) is one of the most common causes of death that kills approximately 17 million people annually. The main reasons behind CVD are myocardial infarction and the failure of the heart to pump blood normally. Doctors could diagnose heart failure (HF) through electronic medical records on the basis of patient's symptoms and clinical laboratory investigations. However, accurate diagnosis of HF requires medical resources and expert practitioners that are not always available, thus making the diagnosing challengeable. Therefore, predicting the patients' condition by using machine learning algorithms is a necessity to save time and efforts. This paper proposed a machine-learning-based approach that distinguishes the most important correlated features amongst patients' electronic clinical records. The SelectKBest function was applied with chi-squared statistical method to determine the most important features, and then feature engineering method has been applied to create new features correlated strongly in order to train machine learning models and obtain promising results. Optimised hyperparameter classification algorithms SVM, KNN, Decision Tree, Random Forest, and Logistic Regression were used to train two different datasets. The first dataset, called Cleveland, consisted of 303 records. The second dataset, which was used for predicting HF, consisted of 299 records. Experimental results showed that the Random Forest algorithm achieved accuracy, precision, recall, and F1 scores of 95%, 97.62%, 95.35%, and 96.47%, respectively, during the test phase for the second dataset. The same algorithm achieved accuracy scores of 100% for the first dataset and 97.68% for the second dataset, while 100% precision, recall, and F1 scores were reached for both datasets.

## 1. Introduction

Cardiovascular disease (CVD) is one of the most common diseases that cause morbidity and mortality. It contributes to a third of deaths worldwide according to the American College [1]. Since 2102, numerous surveys concluded that nearly 56 million people lost their lives in 2012; amongst them, 17.5 million died due to CVD [2]. According to [3], CVD has three types: circulatory, structural, and electrical. In circulatory CVD, which is also called coronary artery disease (CAD), atherosclerosis (i.e., accumulation of plaques) is built up on the inner walls of a coronary artery, causing the arteries to harden [4–6]. This accumulated plaque consists of cholesterol or fatty deposits that restrict blood flow through the arteries. When CAD progresses, potentially fatal symptoms, such as stroke and myocardial infarction, begin to appear.

Therefore, early treatment and recovery of atherosclerosis are important to minimise CVD risks. Several imaging methods are introduced with high accuracy and sensitivity to determine the disease severity [7, 8]. They include dobutamine stress echocardiography, exercise electrocardiogram (ECG), coronary computed tomography angiography, myocardial perfusion scintigraphy, and conventional coronary angiography. However, all these imaging methods could only discover existing atherosclerosis that already developed. For instance, ECG is an easy-to-access diagnostic tool that records the electrical activity of the heart [9]. ECG signals could be obtained during exercise as a patient undergoes stress [10]. ECG signals allow heart rate variability signals to be extracted [11]. The ECG technique is the primary choice for evaluating heart conditions because it is easy to perform, inexpensive, and noninvasive. However, manual diagnosis of ECG signals is tedious and difficult because the signals differ morphologically.

In addition, the discovery of biomarkers, such as chest pain, serum cholesterol, resting electrocardiographic results, resting blood pressure, maximum heart rate, depression, fasting blood sugar, exercise-induced angina, slope of peak exercise, number of major vessels, segment, and thallium stress, in clinical samples has been helpful in understanding and diagnosing atherosclerosis. Therefore, to conduct a diagnostic process of ECG signals with high accuracy, artificial intelligence techniques are used to help diagnose arteriosclerosis through these tests and biomarkers. As the data collected for these biomarkers are huge, most of the studies on the diagnosis systems focused on the preprocessing process to clean the data, select the most important representative features, delete redundant features, and choose appropriate classification algorithms. For instance, Zimmerli et al. presented an assay for polypeptides that contribute to biomarkers for identifying CAD. They screened 359 urine samples from 88 patients with CAD and 282 controls. The system reached a sensitivity of 98% and a specificity of 83% [12]. Likewise, Tan et al. presented three diagnostic algorithms for a set of diagnostic features of heart disease. The systems were evaluated by accuracy, sensitivity, and specificity on four datasets: Cleveland, Hungarian, SPECTF, and Switzerland. Their proposed system reached accuracy scores of 81.19%, 92.68%, 82.7%, and 84.52% for Cleveland, Hungarian, SPECTF, and Switzerland, respectively [13]. Arabasadi et al. presented a hybrid method to diagnose CAD, and their algorithm was able to increase the performance of neural networks by 10% through a genetic algorithm (GA), which optimises primary weights. The system achieved an accuracy of 93.85%, a sensitivity of 97%, and a specificity of 92% [14]. Maji and Arora presented a hybrid method between Decision Tree and ANN classifiers for diagnosing heart disease. The ANN achieved an accuracy of 77.4%, a sensitivity of 77.4%, and a specificity of 21.7% [15]. Saqlain et al. presented three algorithms for selecting the most important features, which are the Fisher score-based algorithm, the algorithm for selecting the most important features based on forward, and the algorithm for selecting the most important features based on the reverse. The selected features were entered into an SVM classifier based on the RBF kernel for the diagnosis of four cardiac disease datasets. The system achieved an accuracy of 81.19% for the Cleveland dataset [16]. Babu et al. applied 14 features that were extracted, then fed into three classification algorithms, namely,*K*-means, MAFI, and Decision Tree, to classify heart disease. All algorithms performed well for diagnosing heart failure [17]. Reddy and Khare presented a rule-based fuzzy logic (RBFL) algorithm to predict heart disease and help medical practitioners diagnose it at an early stage. The locality preserving projection (LPP) method was first applied to determine the most important characteristics of the UCI dataset. The RBFL algorithm achieved an accuracy of 78% [18]. Feshki et al. presented Particle Swarm Optimization method with Neural Network Feed Forward Back Propagation, which reduced the features from 13 features to 8 enhanced features; the system reached an accuracy of 91.94% with these selected features [19]. Uyar and İlhan presented a GA based on a Recurrent Fuzzy Neural Network (RFNN) algorithm trained to diagnose heart disease, and the system achieved an accuracy of 97.78% [20]. Haq et al. presented seven machine learning algorithms to classify features extracted by three methods for selecting features of the heart failure dataset. The performance of the systems was evaluated using several scales such as accuracy, sensitivity, specificity, receiving optimism curves, and AUC, and they reached good results [21]. Kerexeta et al. presented two methods for predicting the risk of returning a patient with high blood pressure back to hospital. In the first method, the supervised and supervised classification methods were combined, and the system reached an AUC of 61%. The second method was combined the Naïve Bayes classifiers and the Decision Tree, and the method achieved an AUC of 73%. The limitations in this study are related to the dataset because the study is based on a readmission day threshold [22]. Adler et al. presented machine learning algorithms that link patient features with mortality, by training a Decision Tree algorithm with a set of features associated with high mortality risk. Eight characteristics that have a very high risk of death were extracted, and the risk score for these advantages was 88% for the AUC scale. Limitation of MARKER-HF was derived from two hospitals, San Diego, California, and is therefore subject to demographic region bias [23]. Jin et al. presented an effective method for predicting heart failure by using a neural network, where they used one-hot encoding and word vectors to model the diagnosis and prediction of heart failure through a long short-term memory algorithm [24]. Gjoreski et al. presented a method that combines machine learning and deep learning to diagnose heart failure based on the heart sounds of 947 people. Machine learning algorithms train expert features, while deep learning models train from the spectral chains of the heart signal. The method achieved an accuracy of 92.9 and an error rate of 7.1% [25]. Vijayashree and Sultana presented the Particle Swarm Optimization (PSO) method, which selects the most appropriate features and increases the important features for diagnosing heart disease. PSO was used in conjunction with SVM to reduce the number of features and increase accuracy; the system achieved good results for diagnosing heart disease [26].

However, most of the discussed studies above are insufficient. Therefore, the main contributions of this paper are as follows:

- Adjust and optimise hyperparameter of five machine learning algorithms for predicting heart failure (HF) with high accuracy
- Select the most important features with strong correlation to obtain more realistic diagnostic results
- Apply feature scoring to rank the features based on the correlated to the target feature
- Solve the class imbalance issue in the second dataset by synthetic minority oversampling (SMOTE) technique
- Create new features that have strong correlation with the target feature to obtain more realistic diagnostic results

The remainder of this study is organised as follows.  Section 2 describes a background on the overview and risk factors of HF diseases and an explanation of machine learning algorithms.  Section 3 discusses the exploratory data analysis (EDA) to describe the two sets of data and explain the correlation between the features and the replacement of missing values.  Section 4 presents data processing that includes subsections for engineering and selection of the most important features.  Section 5 describes the experimental result and discussion part. Finally, Section 6 concludes the paper.

## 2. Background

### 2.1. Overview and Risk Factors of HF Diseases

Heart disease and atherosclerosis are disorders of the heart and arteries that include HF, coronary heart disease (heart attacks), cerebrovascular diseases (strokes), and other types of heart disease [27]. CVD is one of the most common causes of death in the world, with the number of deaths reaching roughly 17 million annually worldwide. HF occurs because the heart is unable to pump enough blood to the rest of the body. It is caused by diabetes, high blood pressure, and other heart diseases [28]. Doctors classify HF into two types on the basis of the ejection fraction value, which is the percentage of blood that the heart pumps during one contraction and a physiological value ranging from 50% to 75%. Low HF causes the ejection fraction, previously called left ventricular (LV) HF, to drop below 40% [29]. The final ejection fraction rate is HF with preserved ejection fraction, previously called diastolic HF, with a normal ejection fraction. In this case, during systole, the LV contracts normally but fails during diastole due to ventricular stiffness; thus, blood pumping is impaired [30]. Due to the importance of the heart organ, HF prediction has become of utmost importance for physicians in predicting HF; however, even today in clinical practices, physicians have failed to reach high accuracy in predicting HF [31]. Electronic medical records could be considered one of the most useful sources for uncovering correlated data amongst patients and an important source for researchers and clinical practices [32]. Machine learning techniques play an important role in analysing medical records, predicting the survival of each patient with HF, and detecting the most important features that lead to HF [33].

### 2.2. Machine Learning

Machine learning is the ability of computer programs to adapt, learn, and address new problems. Machine learning algorithms work on medical diagnostics and help experts support their decisions about their medical diagnosis. Machine learning has the ability to learn from training data and solve classification problems for new data [34].

#### 2.2.1. *K*-Nearest Neighbor (KNN)

KNN is used to solve classification problems based on stored data. The algorithm trains the dataset and stores it in the memory. When the classification process is to test new data points, the algorithm works on the basis of similarity of the state between the new data point and the stored dataset and classifies new data in accordance with the most similar class on the basis of the value of *K* and the closest one on the basis of Euclidean distance.

#### 2.2.2. Support Vector Machine (SVM)

This model is similar to neural networks in its objective of adjusting a set of parameters, which allow to establish boundaries in a dimensional space and approximate functions or separate patterns in different regions of the attribute space. The difference lies in the training method for adjusting the parameters. By contrast, SVMs base their training on maximizing the margin between the hyperplane and the instances of two classes (initially, this model was designed to solve problems of classifying two classes but extensions for multiclass and regression problems exist) [35]. The algorithm works with linear and nonlinear data. When the data are linear, the algorithm finds a hyperplane with maximum margin, which is the largest distance between data points of two classes. Maximum margin gives the algorithm power to classify the test dataset with high confidence. Hyperplane is the decision boundary that separates the class data. Support vectors are the data points that form close to the hyperplane. In accordance with support vectors, the distance is increased to maximize the margin. Thus, the hyperplanes change when removing these support vectors. Therefore, these points build an SVM classifier. For nonlinear data, the original coordinate area is converted into a separable space [35].

#### 2.2.3. Decision Tree

Decision Tree is used to solve classification problems. It consists of root node, inner nodes, branches, and leaf nodes. It is organised in the form of a tree, where the root node represents the complete dataset, the internal nodes represent the features contained in the dataset, the branches represent the decision-making area, and the leaf nodes represent the outcome. Decisions are made on the basis of features selected in the dataset. When predicting dataset features, the algorithm starts from the root node. The algorithm compares the value of the root feature with the feature's values of the dataset, and in accordance with the comparison, it moves to the next nodes. The process continues to the next node, where the feature in the node is compared with the features in the next nodes, and the process continues until the leaf node is obtained.

#### 2.2.4. Random Forest

Random Forest is used to solve classification problems. It works on the basis of ensemble learning, as it solves the problem by combining several classifiers to improve the performance of the algorithm. The algorithm contains several classifiers of Decision Trees. Each Decision Tree works with a subset of data and average taken to improve prediction accuracy. Instead of taking prediction from one tree, the Random Forest algorithm takes prediction from each tree and works on prediction on the basis of majority voting.

#### 2.2.5. Logistic Regression

Logistic Regression is one of the supervised machine learning algorithms used to solve classification problems to predict probability-based target variables. The target or dependent variables are binary variables that contain two classes; multinomial target variables have three or more unordered types or ordinal variables, where the target variable contains three or more ordered variables.

## 3. Exploratory Data Analysis (EDA)

This section focuses on data preprocessing, including missing data treatment, outlier removal, and feature correlation test.  Figure 1 describes the structure applied to evaluate the performance of the algorithms on the two datasets for early diagnosis of heart disease.

### 3.1. Description of Datasets

Two datasets of heart disease and failure data were collected from the UCI machine learning repository. The first dataset is called Cleveland (https://archive.ics.uci.edu/ml/datasets/heart+Disease) [36], which is commonly used by heart-disease diagnostic machine learning researchers. The Cleveland dataset consists of 303 records, with 76 features. However, the UCI repository provides approved 14 features that are most influential in the field of diagnosing heart disease.  Table 1 describes the features, measures, and their ranges. Thirteen features could be used for diagnosing heart disease, and one target feature could be used to describe whether or not a disease exists.

The second dataset for predicting HF contains medical records of 299 patients with HF (https://archive.ics.uci.edu/ml/machine-learning-databases/00519/) [37]. The dataset was collected from the Faisalabad Institute of Heart Disease and the Allied Hospital in Faisalabad.  Table 2 describes the features, measurement, and range of HF prediction. Twelve features could predict HF in addition to the target feature that describes whether or not the patient died during follow-up.  Table 2 also explains each feature and the subsections that represent each feature.

### 3.2. Statistical Feature Correlation Using Heat Map

A heat map is a graphical representation that shows the correlation between features and the percentage of correlation of each feature with the other. It also describes the correlation of all features with the target feature. Statistics is a set of computational tools used to interpret raw data and convert them into information to be understood. It is one of the tools used in the field of machine learning. Statistics and machine learning are two closely related fields. In this study, descriptive statistics were calculated on the dataset of heart disease (Cleveland dataset) and HF to obtain the features of common and correlated data samples as mean, standard deviation, and max and min values.  Table 3 describes the statistical processes applied to the Cleveland dataset, where count refers to the number of features of dataset, mean refers to the mean between the features of the dataset, std refers to the standard deviation between the features of the dataset, and min and max refer to the minimum and maximum values amongst the features of the dataset. Descriptive statistics have a positive effect on graphic visualisations to easily understand raw data and relate the data to one another.  Figure 2 illustrates the correlation between the features of the dataset with one another. “cp” (chest pain), “thalach,” and “slope” features were correlated closely with the target feature, and the correlation of each distinctive with the other was noted.

### 3.3. Treatment of Missing Values

Datasets that contain missing values need to be addressed and cleaned up. Missing values result from patients missing out on some metrics when they undergo a test. The Cleveland dataset contained missing values, and the second dataset contained six missing values. Thus, statistical measures must be applied to replace the missing values. Statistical measures, such as mean, median, and standard deviation, are applied to replace numerical values. The mode method is also applied to replace nominal values.  Table 4 describes the missing features for the Cleveland dataset after processing. The mean method was applied to replace the numerical values by calculating the mean for the features and replacing the missing value. The mode method was also applied to replace the missing nominal values by replacing the nominal value with the most common value in the features.

### 3.4. Balancing a Dataset

With regard to data balancing, the Cleveland dataset contains 165 people with heart disease and 138 people without heart disease. Thus, the dataset is balanced. Regarding the second dataset, the number of people who died during follow-up was 203, while 96 people did not die during follow-up; therefore, the dataset is unbalanced. To obtain satisfactory results, the dataset must be balanced during the training phase. In this study, the synthetic minority oversampling technique (SMOTE) was applied, which is one of the appropriate methods for balancing the dataset. SMOTE technique searches for minority classes and finds the nearest neighbor for each point (value) in the minority class to generate new synthetic samples at a given point randomly, the mechanism continues until the dataset is balanced during the training phase, and the minority class becomes approximately equal to the majority class.  Table 5 describes the second dataset before and after the application of the SMOTE technique, where it is noted that the cases of the minority class (die during follow-up) increased from 79 cases to 160 cases; thus, the two classes became equal during the training phase.

### 3.5. Data Conversion

Data processing is the ability to transform data into useful data that could be manipulated and analysed. In this study, categorical variables were converted into dummy variables, which include the values 0 and 1. Dummy variables are useful for multiple groups in single regression equations.  Table 6 describes the dataset after converting the categorical features to dummy.

### 3.6. Data Standardization

Preprocessing is one of the most important stages of data mining, and it leads to diagnostic accuracy in the following stages. In this study, data standardization method was applied to the two datasets. Standardization coordinates the data internally, ensures that all data have the same formatting and content, and gives the dataset more meaning. It transforms the dataset, in which its distribution has a mean of 0 and a standard deviation value of 1. In this study, the standardization method was applied in accordance with Equation (1) and the dataset obtained its data distribution. Each feature in the dataset obtained its value subtracted from the mean and divided by the standard deviation of the whole dataset.  Table 7 describes the application of the standardization method to four features of the dataset, namely, “trestbps,” “chol,” “thalach,” and “oldpeak.”

(1) $$\begin{array}{c} z=\frac{\;x-\mu }{\sigma }, \end{array}$$

where *x* denotes the value of each feature, *μ* refers to the mean for each feature, *σ* denotes the standard deviation of the dataset, and *z* refers to the features in a standardised form.

## 4. Feature Processing

### 4.1. Feature Engineering

Feature engineering, also called feature creation, is the process of creating new features from the existing dataset for the purpose of training machine learning models and obtaining more reliable results. Usually, the feature engineering process is manual, relying on intuition, field knowledge, and data manipulation. It is also very tedious and limited. Thus, automated feature engineering helps data scientists create new features that are well correlated and use them for training.  Table 8 describes the additional relevant extracted features correlated between two features, in which 60 features from the original Cleveland dataset containing 13 features were obtained. With these new features, the solution to the classification problem could be enhanced. The better the features, the better the results.

### 4.2. Feature Selection

Feature selection methods are aimed at reducing unimportant features and focusing on features that contribute to the most predictable feature of the target feature. Reducing the number of features reduces the computational cost of modelling and improves the performance of the model. The methods for selecting features by means of statistics include assessing the relationship between each feature and the target feature and selecting the input features that have the strongest correlation with the target feature. In this study, SelectKBest with the chi-square method was used to extract the best features from the dataset. The SelectKBest function uses this method as a score function to determine a score and the correlation between each feature and target feature. It passes chi-square to determine the score between each feature and the target feature. If the resulting value is lower, then the feature is independent of the target feature, while higher resulting value indicates that the feature is not randomly related to the target feature.  Table 8 describes how the SelectKBest function automatically returns the first *K* features with the highest scores of the Cleveland dataset. The exang_oldpeak2 feature, which is correlated between exang feature and oldpeak2 feature, had the highest score of 652.85, while the lowest fbs feature score was 0.18.

## 5. Experimental Result and Discussion

### 5.1. Splitting Datasets

The Cleveland dataset consisted of 303 records for two classes: heart disease (class 1), which contained 165 records by 54.46%, and normal (class 0), which contained 138 records by 45.54%. The second dataset (HF) contains 299 records for two classes: died during follow-up (class 1), containing 203 records by 67.87%, and did not die during follow-up (class 0) containing 96 records by 32.13%. After balancing the second dataset, the two classes became equal to 160 cases during the training phase.  Table 9 describes the distribution of the two datasets for the two groups during the training and testing phases.

### 5.2. Evaluation Criteria

Four qualitative measures were used, namely, accuracy, precision, recall, and F1score, to evaluate the proposed systems on the two datasets, as shown in Equations (2)–(5).

(2) $$\begin{array}{c} \text{Accuracy}=\frac{\text{TN}+\text{TP}}{\text{TN}+\text{TP}+\text{FN}+\text{FP}}*100\%, \end{array}$$

(3) $$\begin{array}{c} \text{Precision}=\frac{\text{TP}}{\text{TP}+\text{FP}}*100\%, \end{array}$$

(4) $$\begin{array}{c} \text{Recall}=\frac{\text{TP}}{\text{TP}+\text{FN}}*100\%, \end{array}$$

(5) $$\begin{array}{c} \text{F}1\text{ score}=2*\frac{\text{Precision}*\text{recall }}{\text{Precision}+\text{recall }}*100, \end{array}$$

where TP is the number of heart disease samples that are correctly classified, TN is the number of nonheart disease samples that are correctly classified, FN is the number of heart disease samples classified as nonheart disease, and FP is the number of nonheart disease samples classified as heart disease [38].

### 5.3. Results for the Cleveland Dataset

Several machine learning algorithms have been applied to predict heart disease for patient survival. Classification and hyperparameter algorithms that produce optimal networks have been optimised to reduce function loss and to obtain high diagnostic performance. Tuning hyperparameter is an important process for determining the behaviour of machine learning networks during training. In this study, machine learning models were applied to the dataset containing 13 original features of 303 patients. New features were created through the correlation of the original features, and they were expanded to 60 features for each patient. The dataset was divided randomly into 80% for training (242 patients) and 20% for testing (61 patients).  Figure 3 shows the performance of classification algorithms on the dataset during the training and testing phases.  Table 10 shows the diagnostic results for heart disease by using five machine learning algorithms during the training and testing processes. During the training phase, Decision Tree and Random Forest obtained the best results of 100% for all measures. However, during the testing phase, SVM and KNN algorithms achieved the best results, with an approximate rate of 90% for all measures. Logistic Regression obtained the lowest result during the training and testing phases amongst all the algorithms. During the training phase, SVM, KNN, Decision Tree, Random Forest, and Logistic Regression reached accuracy scores of 92.56%, 87.60%, 100%, 100%, and 87.60%, respectively; in the testing phase, their accuracy scores were 90.16%, 90.16%, 81.97%, 85.25%, and 88.52%, respectively. For the precision, during the training phase, SVM, KNN, Decision Tree, Random Forest, and Logistic Regression reached of 93.45%, 88.82%, 100%, 100%, and 88.19%, respectively; in the testing phase, their precision rates were 90.12%, 90.26%, 82.43%, 85.82%, and 88.56%, respectively. During the training phase, SVM, KNN, Decision Tree, Random Forest, and Logistic Regression reached recall rates of 92.52%, 87.63%, 100%, 100%, and 87.44%, respectively; in the testing phase, their recall rates were 90.45%, 90.38%, 82.39%, 85.29%, and 89.46%, respectively. For the F1 score, during the training phase, SVM, KNN, Decision Tree, Random Forest, and Logistic Regression reached 92.98%, 88.23%, 100%, 100%, and 87.81%, respectively; In the testing phase, their F1 scores were 90.28%, 90.32%, 82.41%, 85.55%, and 89%, respectively.

Table 11 and Figure 4 describe the analysis of the results obtained in depth at each class, where heart disease = 1 and nonheart disease = 0. The dataset was divided into 80% for training and 20% for testing. The training data were further divided into 133 for heart disease and 109 for nonheart disease, while the test data were divided into 32 for heart disease and 29 for nonheart disease. During the training phase, Decision Tree and Random Forest achieved the best results for diagnosing heart and nonheart diseases by 100% for all measures. However, during the testing phase, KNN achieved better than the rest of the algorithms, with rates of 90% for all criteria when diagnosing negative cases (nonheart disease) and 91% for all criteria when diagnosing positive cases (heart disease). First, in the analysis and interpretation of the results of the diagnosis of heart disease (class 1) during the training phase, SVM, KNN, Decision Tree, Random Forest, and Logistic Regression reached a precision of 92%, 88%, 100%, 100%, and 87%, respectively; in the testing phase, their precision was 93%, 91%, 86%, 87%, and 90%, respectively. For the recall, during the training phase, SVM, KNN, Decision Tree, Random Forest, and Logistic Regression reached a recall of 95%, 90%, 100%, 100%, and 91%, respectively; in the testing phase, their recall was 88%, 91%, 78%, 84%, and 88%, respectively, while for the F1 score during the training phase, SVM, KNN, Decision Tree, Random Forest, and Logistic Regression reached a recall of 93%, 89%, 100%, 100%, and 89%, respectively; in the testing phase, their F1 scores were 90%, 91%, 82%, 86%, and 89%, respectively. Second, in the analysis and interpretation of the results of the diagnosis of nonheart disease (class 0) during the training phase, SVM, KNN, Decision Tree, Random Forest, and Logistic Regression reached a precision of 93%, 88%, 100%, 100%, and 88%, respectively; in the testing phase, their precision was 87%, 90%, 78%, 83%, and 87%, respectively. For the recall, during the training phase, SVM, KNN, Decision Tree, Random Forest, and Logistic Regression reached a recall of 90%, 84%, 100%, 100%, and 83%, respectively; in the testing phase, their recall was 93%, 90%, 86%, 86%, and 90%, respectively, while for the F1 score during the training phase, SVM, KNN, Decision Tree, Random Forest, and Logistic Regression reached a recall of 92%, 86%, 100%, 100%, and 86%, respectively; in the testing phase, their F1 scores were 90%, 90%, 82%, 85%, and 88%, respectively.

### 5.4. Results of HF Dataset

A medical dataset containing 299 patients with HF was analysed. This section describes the outcomes that predicted patient survival during the follow-up period. The features were arranged in accordance with the correlation with the target feature (death event), and the data lost due to the loss of some tests during patient examination were processed and replaced. Correlated features were created between two features, and they have an effective effect on increasing the accuracy of prediction. Hyperparameter classification algorithms were adjusted to reduce the loss function and obtain high predictive results. The dataset was divided into 80% for training (160 patients died during follow-up, and 79 patients did not die during follow-up) and 20% for testing (43 patients died during follow-up, and 17 patients did not die during follow-up).  Figure 5 illustrates the evaluation of the dataset on the performance of the algorithms during the training and testing phases.  Table 12 shows the results for predicting HF by using five classification algorithms during the training and testing phases. Random Forest achieved the best performance during both phases, followed by Decision Tree, KNN, SVM, and Logistic Regression. During the training phase, SVM, KNN, Decision Tree, Random Forest, and Logistic Regression reached an accuracy of 92.35%, 96.82%, 96.46%, 97.68%, and 91.05%, respectively; in the testing phase, their accuracy was 90%, 93.33%, 95%, 95%, and 88.33%, respectively. For the precision, during the training phase, SVM, KNN, Decision Tree, Random Forest, and Logistic Regression reached of 95.41%, 95.76%, 97.11%, 100%, and 94.52%, respectively; in the testing phase, their precision rates were 93.02%, 93.33%, 93.48%, 97.62%, and 93%, respectively. During the training phase, SVM, KNN, Decision Tree, Random Forest, and Logistic Regression reached recall rates of 96.10%, 98.51%, 100%, 100%, and 92.39%, respectively; in the testing phase, their recall rates were 93.02%, 97.67%, 100%, 95.35%, and 90%, respectively. For the F1 score, during the training phase, SVM, KNN, Decision Tree, Random Forest, and Logistic Regression reached 95.75%, 97.12%, 98.53%, 100%, and 93.44%, respectively; in the testing phase, their F1 scores were 93.02%, 95.45%, 96.63%, 96.47%, and 91.93%, respectively.

Table 13 and Figure 6 describe the HF results predicted using the five machine learning algorithms for each class (1 = died during follow-up and 0 = did not die during follow-up). The training data were divided into 160 for class 1 and 79 for class 0, while the test data were divided into 43 for class 1 and 17 for class 0. Random Forest achieved the best result during the training phase for both classes, with 100% for each criterion (precision, recall, and F1 score). During the testing phase, Random Forest also achieved the best precision for predicting HF, with 97% for class 1 and 98% for class 0. Meanwhile, Decision Tree achieved the best recall of 100% for both classes. Random Forest showed the best F1 score of 96% for predicting positive cases and 97% for predicting negative cases. First, in the analysis and interpretation of the results of the diagnosis of died during follow-up (class 1) during the training phase, SVM, KNN, Decision Tree, Random Forest, and Logistic Regression reached a precision of 93%, 91%, 98%, 100%, and 96%, respectively; in the testing phase, their precision was 94%, 94%, 94%, 97%, and 93%, respectively. For the recall, during the training phase, SVM, KNN, Decision Tree, Random Forest, and Logistic Regression reached a recall of 96%, 99%, 100%, 100%, and 91%, respectively; in the testing phase, their recall was 94%, 98%, 100%, 95%, and 92%, respectively, while for the F1 score during the training phase, SVM, KNN, Decision Tree, Random Forest, and Logistic Regression reached a recall of 97%, 98%, 99%, 100%, and 93%, respectively; in the testing phase, their F1 scores were 94%, 96%, 97%, 96%, and 93%, respectively. Second, in the analysis and interpretation of the results of the diagnosis of did not die during follow-up (class 0) during the training phase, SVM, KNN, Decision Tree, Random Forest, and Logistic Regression reached a precision of 92%, 89%, 97%, 100%, and 94%, respectively; in the testing phase, their precision was 92%, 92%, 92%, 98%, and 93%, respectively. For the recall, during the training phase, SVM, KNN, Decision Tree, Random Forest, and Logistic Regression reached a recall of 95%, 97%, 100%, 100%, and 93%, respectively; in the testing phase, their recall was 91%, 97%, 100%, 96%, and 90%, respectively, while for the F1 score during the training phase, SVM, KNN, Decision Tree, Random Forest, and Logistic Regression reached a recall of 95%, 96%, 98%, 100%, and 94%, respectively; in the testing phase, their F1 scores were 92%, 94%, 95%, 97%, and 91%, respectively.

### 5.5. Comparison of the Performance of Algorithms between the Two Datasets

Similar data processing methods, preprocessing, processing features and arranging them in order of importance, and classification algorithms, were applied to the two datasets, Cleveland and HF datasets. Through the analyses in the previous sections, the diagnostic systems were able to evaluate the HF dataset, with an accuracy that exceeded the evaluation of the Cleveland dataset during the test phase.  Table 14 and Figure 7 describe the analytical results to compare the performance of machine learning algorithms on the two datasets. First, the performance of the SVM, KNN, Decision Tree, Random Forest, and Logistic Regression on the Cleveland dataset during the training phase reached to an accuracy of 92.56%, 87.60%, 100%, 100%, and 87.60%, respectively; in the testing phase, their accuracy was 90.16%, 90.16%, 81.97%, 85.25%, and 88.52%, respectively. Second, the performance of the SVM, KNN, Decision Tree, Random Forest, and Logistic Regression on the HF dataset during the training phase reached to an accuracy of 92.35%, 96.82%, 96.46%, 97.68%, and 91.05%, respectively; in the testing phase, their accuracy was 90%, 93.33%, 95%, 95%, and 88.33%, respectively.

### 5.6. Comparison with Previous Studies

Table 15 and Figure 8 describe the evaluation of machine learning network models proposed by several criteria evaluated in relevant previous studies. As noted, previous studies were evaluated with some criteria. All previous studies reached an accuracy ranging between 93.85% and 77.55%, while the accuracy of the proposed system reached 100% during training and 95% during testing. The previous studies reached a precision ranging between 91.4% and 77.4%, while the proposed system reached 100% during training and 97.62% during testing. The recall (sensitivity) in previous studies reached a rate ranging between 97% and 72%, while the proposed system reached 100% during training and 95.35% during testing.

## 6. Conclusion and Future Work

The importance of electronic biometrics was verified in the process of predicting heart disease and failure. The SelectKBest function with the chi-square statistical method was applied to select the features with strong correlation with the target feature, and then, the degree between each feature and the target feature was determined. Feature engineering method was also applied to increase the number of correlated features between them and train machine learning models to obtain reliable results that were better than the results obtained from the original features of the two datasets. Machine learning algorithms used optimised hyperparameters and fed them with new features. All algorithms reached superior results during the training and testing phases of the two datasets. During the testing phase, all algorithms achieved better results for the second dataset (HF) than for the first dataset (Cleveland). For the first dataset, Random Forest and Decision Tree reached the best results during the training phase, with 100% for all measures. During the testing phase, SVM and KNN achieved better results than the rest of the algorithms. For the second dataset, Random Forest obtained the best results during both phases. There are some limitations to the study. First, the two datasets used and publicly available are relatively small. Second, the two datasets do not contain feature natriuretic peptides (NPs) which are biomarkers of heart failure, where NPs rise with age and NPs decrease in obese patients. Third, the two datasets did not include advantages about the patients' diet. However, despite the limitations, the two datasets had sufficient features. Our aim was to rank the significance of the features on the basis of the score and correlation feature of heart failure. The future scope of this work is the application of the Internet of Things and the testing of new samples in real time.

## Figures and Tables

**Figure 1:** Experimental methodology of heart disease.

**Figure 2:** Feature correlation of the Cleveland dataset by using heat map.

**Figure 3:** Evaluating the performance of five classifiers on the Cleveland dataset.

**Figure 4:** The performance of classification algorithms for each class.

**Figure 5:** Evaluating the performance of five classifiers on the heart failure dataset.

**Figure 6:** The performance of classification algorithms for each class.

**Figure 7:** Comparison of system performance on the diagnostic accuracy in two datasets.

**Figure 8:** The performance of our systems with the previous studies.

**Table 1:** Diagnosing heart disease features with metrics from the Cleveland dataset.

Features	Description	Explanation	Type
Age	Patient age	Age of patient in year	Numeric
Sex		1 = male	Nominal
	Patient gender	0 = female	
cp		1 = typical angina	Nominal
	Chest pain	2 = atypical angina	
		3 = nonanginal pain	
		4 = asymptomatic	
trestbps	Patient's blood pressure at rest (mm/Hg)	Resting blood pressure (mm/Hg)	Numeric
chol	Patient's cholesterol (mg/dL)	Serum cholesterol (mg/dL)	Numeric
fbs		1 = Fasting blood sugar > 120 mg/dL	Nominal
	Patient's blood sugar during fasting	0 = Fasting blood sugar < 120 mg/dL	
restecg		0 = normal	Nominal
	Electrocardiographic measurement at rest	1 = ST-T wave abnormality	
		2 = probable left ventricular hypertrophy	
thalach	Maximum heart rates	Maximum heart rate achieved	Numeric
exang	Angina due to exercise	1 = exercise induced angina	Nominal
		0 = exercise induced no angina	
Oldpeak	ST depression	ST depression induced by exercise relative to rest	Numeric
Slope		1 = upsloping	Nominal
	Slope of ST	2 = flat	
		3 = downsloping	
ca	Number of major vessels	Number of major vessels (0-3) colored by fluoroscopy	Numeric
thal		3 = normal	Nominal
	Blood disorder	6 = fixed defect	
		7 = reversible defect	
Target		0 = normal	Nominal
		1 = heart disease	

**Table 2:** Heart failure features with metrics from the Allied Hospital dataset.

Features	Explanation	Range	Measurement
Age	Age of patient in year	[40, ..., 95]	Year
Anaemia	1 = haematocrit levels lower than 36%	0, 1	Boolean
	0 = haematocrit levels higher than 36%		
High blood pressure	1 = patient has hypertension	0, 1	Boolean
	0 = patient has no hypertension		
Creatinine phosphokinase	Level of CPK in blood	[23, ..., 7861]	mcg/L
Diabetes	1 = patient has diabetes	0, 1	Boolean
	0 = patient has no diabetes		
Sex	1 = male	0, 1	Boolean
	0 = female		
Platelets	Blood platelets	[25.01, ..., 850.00]	Kiloplatelets/mL
Serum creatinine	Level of creatinine in blood	mg/dL	[0.50, ..., 9.40]
Serum sodium	Level of sodium in blood	mEq/L	[114, ..., 148]
Smoking	1 = patient smokes	0, 1	Boolean
	0 = patient does not smoke		
Time	Periodic follow-up of patient	Days	[4,..., 285]
Death event (target)	1 = patient died during follow-up	0, 1	Boolean
	0 = patient did not die during follow-up		

mcg/L refers to micrograms per litre. mL refers to microlitre. mEq/L refers to milliequivalents per litre.

**Table 3:** Statistical operations for the Cleveland dataset.

Statistical	Age	Sex	cp	trestbps	chol	fbs	restecg	thalach	exang	Oldpeak	Slope	ca	thal	Target
Count	303	303	303	303	303	303	303	303	303	303	303	303	303	303
Mean	54.37	0.68	0.97	131.6	246.3	0.15	0.53	149.7	0.33	1.04	1.4	0.73	2.31	0.54
std	9.08	0.47	1.03	17.54	51.83	0.36	0.53	22.91	0.47	1.16	0.62	1.02	0.61	0.5
Min	29	0	0	94	126	0	0	71	0	0	0	0	0	0
Max	77	1	3	200	564	1	2	202	1	6.2	2	4	3	1

**Table 4:** Missing values.

Features	Missing values
Age	0
Sex	0
cp	0
trestbps	0
chol	0
fbs	0
restecg	0
thalach	0
exang	0
Oldpeak	0
Slope	0
ca	0
thal	0
Target	0
dtype: int64	0

**Table 5:** Balancing the dataset by SMOTE.

	Dataset			
Phase	Training 80%		Testing 20%	
Classes	Did not die during follow-up	Die during follow-up	Did not die during follow-up	Die during follow-up
Before Oversampling	160	79	43	17
After Oversampling	160	160	43	17

**Table 6:** Converting categorical data to dummy.

Age	trestbps	chol	thalach	Oldpeak	Target	Sex_0	Sex_1	cp_0	cp_1	...	Slope_2	ca_0	ca_1	ca_2	ca_3
0	63	145	233	150	2.3	1	0	1	0	0	...	0	1	0	0
1	37	130	250	187	3.5	1	0	1	0	0	...	0	1	0	0
2	41	130	204	172	1.4	1	1	0	0	1	...	1	1	0	0
3	56	120	236	178	0.8	1	0	1	0	1	...	1	1	0	0
4	57	120	354	163	0.6	1	1	0	1	0	...	1	1	0	0

**Table 7:** Preprocessing of data by using standardization method.

	Age	trestbps	chol	thalach	Oldpeak
0	0.95	0.76	−0.26	0.02	1.09
1	−1.92	−0.09	0.07	1.63	2.12
2	−1.47	−0.09	−0.82	0.98	0.31
3	0.18	−0.66	−0.2	1.24	−0.21
4	0.29	−0.66	2.08	0.58	−0.38

**Table 8:** Creation of features and arranging the best features.

No	Feature	Score
1	exang_oldpeak2	652.854396
2	exang_ca	263.212119
3	Sex_oldpeak2	252.657949
4	thal_oldpeak2	247.914913
5	exang_trestbps2	241.749732
6	Thalach	186.180286
7	Oldpeak2	171.4864
8	fbs_oldpeak2	164.89897
9	Age2_oldpeak2	139.151372
10	exang_chol2	131.365522
11	thal_trestbps2	116.88462
12	thal_chol2	113.985724
13	thal_ca	90.668503
14	Sex_trestbps2	78.162433
15	Sex_ca	77.302537
16	Oldpeak	71.692782
17	Ca	71.020719
18	Cp	62.116086
19	Age2_ca	54.956199
20	Age2_trestbps2	53.221349
21	restecg_cp	51.837075
22	fbs_ca	43.441045
23	exang	38.518849
24	Age2_chol2	36.438097
25	Sex_chol2	35.823916
26	fbs_cp	32.072291
27	restecg_thalach2	29.718076
28	exang_thalach2	27.279766
29	Age	22.210517
30	Chol	21.690747
31	exang_slope	20.48139
32	exang_cp	18.443334
33	restecg_slope	18.246965
34	trestbps	15.094591
35	restecg_trestbps2	12.462827
36	thal_thalach2	12.403249
37	Slope	9.677715
38	restecg_oldpeak2	8.249627
39	Sex	7.72169
40	thal_slope	7.199342
41	Sex_thalach2	5.89906
42	fbs_trestbps2	5.897746
43	thal_cp	5.838268
44	Thal	5.75303
45	thalach2	5.688919
46	restecg_chol2	5.639162
47	fbs_slope	5.480661
48	Age2_thalach2	5.466855
49	fbs_thalach2	4.64652
50	Age2_slope	4.031292
51	Sex_slope	2.987813
52	restecg	2.877743
53	Age2_cp	2.324974
54	fbs_chol2	2.116344
55	Age2	2.00334
56	trestbps2	1.655964
57	chol2	0.877493
58	Sex_cp	0.564425
59	restecg_ca	0.256374
60	fbs	0.184946

**Table 9:** Splitting the datasets.

Dataset	Cleveland dataset		HF dataset	
Class	Heart disease	Normal	Died during follow-up	Did not die during follow-up
Training	133	109	160	160
Testing	32	29	43	17

**Table 10:** Results of diagnosing heart disease (Cleveland dataset) by using five machine learning algorithms.

Classifiers	SVM		KNN		Decision Tree		Random Forest		Logistic Regression	
Criteria	Training 80%	Testing 20%	Training 80%	Testing 20%	Training 80%	Testing 20%	Training 80%	Testing 20%	Training 80%	Testing 20%
Accuracy (%)	92.56	90.16	87.60	90.16	100	81.97	100	85.25	87.60	88.52
Precision (%)	93.45	90.12	88.82	90.26	100	82.43	100	85.82	88.19	88.56
Recall (%)	92.52	90.45	87.63	90.38	100	82.39	100	85.29	87.44	89.46
F1 score	92.98	90.28	88.23	90.32	100	82.41	100	85.55	87.81	89.00

**Table 11:** Results of diagnosing heart disease as the category using five machine learning algorithms.

SN	Classifiers	Division of data	Class	Precision (%)	Recall (%)	F1 score (%)	Number of patients
1	SVM	Training (80%)	0	93	90	92	109
2			1	92	95	93	133
3		Testing (20%)	0	87	93	90	29
4			1	93	88	90	32
5	KNN	Training (80%)	0	88	84	86	109
6			1	88	90	89	133
7		Testing (20%)	0	90	90	90	29
8			1	91	91	91	32
9	Decision Tree	Training (80%)	0	100	100	100	109
10			1	100	100	100	133
11		Testing (20%)	0	78	86	82	29
12			1	86	78	82	32
13	Random Forest	Training (80%)	0	100	100	100	109
14			1	100	100	100	133
15		Testing (20%)	0	83	86	85	29
16			1	87	84	86	32
17	Logistic Regression	Training (80%)	0	88	83	86	109
18			1	87	91	89	133
19		Testing (20%)	0	87	90	88	29
20			1	90	88	89	32

**Table 12:** Prediction results of heart failure by using five machine learning algorithms.

Classifiers	SVM		KNN		Decision Tree		Random Forest		Logistic Regression	
Criteria	Training 80%	Testing 20%	Training 80%	Testing 20%	Training 80%	Testing 20%	Training 80%	Testing 20%	Training 80%	Testing 20%
Accuracy (%)	92.35	90.00	96.82	93.33	96.46	95.00	97.68	95.00	91.05	88.33
Precision (%)	95.41	93.02	95.76	93.33	97.11	93.48	100.00	97.62	94.52	93.00
Recall (%)	96.10	93.02	98.51	97.67	100.00	100.00	100.00	95.35	92.39	90.90
F1 score	95.75	93.02	97.12	95.45	98.53	96.63	100.00	96.47	93.44	91.93

**Table 13:** Result prediction of heart failure as the category using five machine learning algorithms.

SN	Classifiers	Division of data	Class	Precision (%)	Recall (%)	F1 score (%)	Number of patients
1	SVM	Training (80%)	0	92	95	95	79
2			1	93	96	97	160
3		Testing (20%)	0	92	91	92	17
4			1	94	94	94	43
5	KNN	Training (80%)	0	89	97	96	79
6			1	91	99	98	160
7		Testing (20%)	0	92	97	94	17
8			1	94	98	96	43
9	Decision Tree	Training (80%)	0	97	100	98	79
10			1	98	100	99	160
11		Testing (20%)	0	92	100	95	17
12			1	94	100	97	43
13	Random Forest	Training (80%)	0	100	100	100	79
14			1	100	100	100	160
15		Testing (20%)	0	98	96	97	17
16			1	97	95	96	43
17	Logistic Regression	Training (80%)	0	94	93	94	79
18			1	96	91	93	160
19		Testing (20%)	0	93	90	91	17
20			1	93	92	93	43

**Table 14:** Accuracy of diagnosing two dataset using five machine learning algorithms.

Dataset	SVM		KNN		Decision Tree		Random Forest		Logistic Regression	
Dataset	Training	Testing	Training	Testing	Training	Testing	Training	Testing	Training	Testing
Cleveland	92.56	90.16	87.60	90.16	100	81.97	100	85.25	87.60	88.52
HF	92.35	90.00	96.82	93.33	96.46	95.00	97.68	95.00	91.05	88.33

**Table 15:** Comparison of the performance between the proposed system and previous studies.

Previous studies	Accuracy (%)	Precision (%)	Recall (%)	F1 score (%)
Arabasadi et al. [14]	93.85	—	97	—
Maji and Arora [15]	77.4	—	77.4	—
Reddy et al. [39]	90	—	91	—
Amin et al. [40]	78.15	78.15	—	80.25
Feshki and Shijani [19]	91.94	91.9	93	—
Pouriyeh et al. [41]	77.55	77.4	83	80.1
Chicco and Jurman [42]	83.8	—	72	71.9
Proposed model first dataset for training	97.68	100	100	100
Proposed model second dataset for training	100	100	100	100
Proposed model first dataset for testing	90.16	90.26	90.38	90.32
Proposed model second dataset for testing	95	97.62	95.35	96.47

## Data Availability

The data used to support the findings of this study were collected from a UCI Machine Learning Repository, in the below links: https://archive.ics.uci.edu/ml/datasets/heart+Disease and https://archive.ics.uci.edu/ml/machine-learning-databases/00519/.
